# Simulation of Transmission System of Crawler Self-propelled Rotary Tiller Based on Deep Learning

This article has been retracted.

**DOI:** 10.1155/2022/6078223

**Published:** 2022-07-30

**Authors:** Luofa Wu, Yanqi Wu

**Affiliations:** ^1^Institute of Agricultural Engineering, Jiangxi Academy of Agricultural Sciences, Nanchang 330200, Jiangxi, China; ^2^Jiangxi Intelligent Agricultural Machinery Equipment Engineering Research Center, Nanchang 330200, Jiangxi, China; ^3^Department of Electronic Engineering, Eindhoven University of Technology, Eindhoven, Netherlands

## Abstract

Because of its good performance, crawler-type running gear plays a very important role in the fields of modern agriculture. This article aims to study the construction of the drive system of the crawler self-propelled rotary tiller with the deep learning network and carry out the system simulation experiment. In this article, deep learning-related algorithms, auto-encoding networks, convolutional neural networks, and structural design of crawler self-propelled rotary tillers are proposed. It then used the self-developed crawler-type rotary tiller and straw paddle machine to compare the field operation performance with the combination of ordinary wheeled tractors and rotary tillers. The experimental results show that the tillage performance indicators such as the working depth, tillage depth stability, ground flatness, stubble pressing depth, and vegetation coverage qualification rate of the “crawler self-propelled tractor + straw stubble pulper” are better than those of “wheel tractor + ordinary rotary tiller” and “crawler tractor + ordinary rotary tiller,” increased by 9.92% and 4.88%, 4.31% and 4.13%, 42.59% and 19.12%, 40.15% and 34.57%, and 13.04% and 7.16%, respectively. The mechanical transplanting index was significantly better than other treatments. The yield increase effect of the field test is remarkable, with the average yield increase rate of 9.63% and 4.57%, which is suitable for popularization and application in the southern double-cropping rice area.

## 1. Introduction

After entering the 21st century, the coordination of weapon equipment and hardware has become a mode of knowledge progress. For the design of hardware, it should also adopt its usual improvement mode and update ideas. As long as it makes full use of the cutting-edge professional hints and logical exploration results, it can always understand the subjective turning of events and the jumps in the design and equipment display and understand the basic goals of improved motorization and informatization. Because of its good performance, crawler-type running gear plays a very important role in the fields of modern agriculture.

For a long time, the development and manufacture of rotary tiller in China have been carried out in accordance with the traditional model of complete machine design, prototype trial production, test analysis, prototype improvement, and product manufacturing. With the increasing development of rotary tiller in China and the maturity of technology, large-scale and lightweight have gradually become the development trend in crawler rotary tiller. The structure of crawler rotary tiller is also becoming more and more complex. The traditional design and development model based on prototype test is not particularly suitable for the research and development and innovation of the Chinese rotary tiller due to its long research and development cycle and large capital investment. In recent years, with the rise and development of virtual prototype technology, there is a new model for the design and development of construction machinery. Compared with the traditional design mode, the dynamic simulation of the virtual prototype can find some problems and make improvements in the design stage by analyzing the force of the main components and performing finite element analysis on some key components. Therefore, the design is more rationalized, the design cycle is shortened, the design cost is saved, and the designed products have greater market competitiveness. For the research of crawler self-propelled rotary tiller, the traditional methods are mostly based on empirical formulas and experiments. It not only has a long development cycle but also is time-consuming and labor-intensive. It is difficult to analyze the performance of rotary tiller. The working environment of the crawler self-propelled rotary tiller is changeable and harsh. It is necessary to use virtual prototyping technology to conduct multi-body dynamic simulation and analysis. In this way, the deficiencies and defects of the traditional design method are well compensated.

The innovation of this article is that the application of a deep learning network to construct the simulation experiment of the transmission system of the crawler self-propelled rotary tiller has certain innovation and practicability. It provides certain technical support for the development of crawler self-propelled rotary tiller transmission. The crawler bulldozer has a complex structure and a changeable and harsh working environment. The virtual prototyping technology is used to conduct multi-body dynamic simulation and analysis.

## 2. Related Works

In recent years, the construction of deep neural network models has become a research hotspot. Many scholars have used deep neural network models in various researches. Litjens et al. audited the vitally profound learning ideas connected with clinical picture examination, reviewing the use of profound learning in picture characterization and different errands [1]. Chen et al. proposed another profound learning structure to intertwine these two highlights, from which the most noteworthy order exactness can be acquired [2]. Kermany et al. had built a significant learning framework-based characteristic instrument for screening patients with ordinary treatable blinding retinal contaminations [3]. Oshea T proposed and examined a few new utilizations of profound learning at the actual layer. By deciphering the correspondence framework as an autoencoder, an essentially new methodology is fostered that treats the correspondence framework plan as a start-to-finish reproduction task [4]. Ravi and Wong introduced a thorough cutting-edge survey of exploration involving profound learning in well-being informatics, giving a vital examination of the relative benefits, possible entanglements of the method as well as its future possibilities [5]. Schirrmeister et al. applied convolutional brain organizations (ConvNets) to the errand of separating among obsessive and ordinary EEG accounts in the Temple University Hospital EEG anomaly corpus [6]. Hou et al. concentrated on the most proficient method to indiscriminately survey the visual nature of pictures by learning rules in language portrayals and proposed a visually impaired IQA model [7]. Zhu et al. broke down the difficulties of involving profound learning in remote detecting information examination and gave assets. Ideally, these assets will make profound learning in remote detecting absurdly simple [8]. The downside of these studies, however, is that the considerations are not comprehensive enough to adapt to more complex situations, and precision needs to be improved.

## 3. Deep Learning Methods

### 3.1. Overview of Deep Learning Methods

#### 3.1.1. Introduction to Deep Learning

Profound learning (DL) is an extremely famous strategy in AI, covering a wide scope of hypothetical viewpoints. To accomplish more astute human-PC collaboration, specialists impersonate the human cerebrum and thinking and lay out different brain network models [9, 10]. Profound learning is one of them [11]. DL is a staggered portrayal learning technique that learns information highlights by making models. Finding a superior information portrayal is the basic role of portrayal learning [12, 13]. As displayed in Figure 1, the construction of each layer of the profound learning strategy is the same as the conventional brain network structure, including the info layer, the secret layer, and the result layer, yet the profound learning technique has a more profound design and more grounded ability to learn. Its essence is to achieve high-dimensional feature representation by stacking multiple hidden layers and complex network structure models, supplemented by a large number of sample data for training, to adjust the weights in the deep network.

As shown in Figure 1, by connecting multiple network layer structures, the output of the upper layer is used as the input of the lower layer, and the hierarchical expression of the input data is realized. The training method is generally to use the backpropagation (BP) algorithm or its variants to update the weights. The resulting deep network model is called a deep neural network (DNN).

Profound growing experiences are non-direct. The handled information can be either discourse, pictures, text, etc., and can be gained from low-level to undeniable-level unique highlights. The educational experience can be either managed or unaided. Among the techniques for profound learning, convolutional brain network is a sort of regulated learning.

(1) Unsupervised deep learning algorithm
  1. Autoencoder. Autoencoder is an unaided learning calculation that embraces back proliferation calculation and is utilized for high-layered complex information handling or element extraction. The autoencoder is a three-layer brain organization, the first and third layers are the info layer and the result layer separately, and the center layer is the secret layer for including extraction of the information obtained by the primary layer.  Figure 2 is an autoencoder training flow chart.
  2. Restricted Boltzmann Machines. Limited Boltzmann machines are haphazardly created irregular organizations that gain likelihood conveyances from an information dataset. The neurons of the confined Boltzmann machine are irregular, or, at least, there are just two result states (dynamic and dormant), which are generally addressed by 0 and 1 in double.  Figure 3 is a structural diagram of a restricted Boltzmann machine.
(2) Supervised Deep Learning Algorithms. The fundamental contrast among directed and solo learning is that managed learning has another name than unaided discovering that can address the idea of the information [14]. Managed learning is additionally separated into two classes: relapse examination and arrangement. In relapse examination, it is partitioned into different sorts as per the number of autonomous factors, subordinate factors, and the connection between them. Relapse strategies are summed up as LR models for multi-order issues. Softmax relapse is in many cases utilized as the last classifier layer in managed profound learning [15]. Coming up next is a point-by-point acquaintance from Softmax with convolutional neural networks.
  1. Softmax Classifier. Prior to presenting Softmax relapse, presenting calculated regression is fundamental. Calculated relapse is a straightforward double characterization calculation. One of the more important formulas in logistic regression is the step function: *Q*(*X*)=1/1+*E*^−*θ*^*Z*^*X*^, its waveform is shown in Figure 4, and the value range is between [0,1]. Figure 4 is the logistic regression step function formula [16].
  2. Convolutional Neural Network. A convolutional neural network (CNN) is one of the DL network structures. Its trademark is that the organization structure contains countless convolution tasks. Furthermore, actuation works and pooling layers are likewise its fundamental designs. These three fundamental designs cause it to have better neighborhood discernment attributes and element deliberation capacity than multi-layer perceptron (MLP) [17]. As of now, CNN has been broadly utilized in numerous region fields of picture handling and PC vision, for example picture characterization, picture semantic division, and visual article recognition [18, 19].

Figure 5 is a representation of the CNN network structure. In the figure, the mitotic image is inputted and decomposed into three channels into the network. The C layer and the S layer in the network model represent the convolution layer and the pooling layer, respectively. First, the feature map is obtained in the C1 layer by convolution, and then the feature map is pooled in the C2 layer. By analogy, the final connection becomes a vector, and the final recognition result is obtained through the traditional artificial neural network algorithm. Among them, the convolution operation and the pooling operation are obtained by updating the weights, adding thresholds, and activating the activation function to obtain the output node of this layer.

The preparation of convolutional brain networks is managed. The general course of boundary preparing is: inputting information, forwarding proliferation layer by layer, and acquiring the organization result of each layer. As indicated by the contrast between the genuine real result and the normal result of the organization, the BP calculation is utilized to conversely change the mistake and update the organization boundaries [20]. The preparation interaction of the completely associated layer incorporates computation yield, back proliferation, and weight update.

(a) Calculate the output
For the *l* layer of the totally related layer, the outcome is
  (1) $$\begin{array}{c} \left\{\begin{array}{c} A^{x}=g\left(W^{x}\right)\\ C^{x}=T^{x}A^{x-1}+P \end{array}\right.,\\ E^{\text{d}}=\frac{1}{2}\overset{l}{\underset{k=1}{\sum }}{\left(S_{k}^{\text{d}}-B_{k}^{\text{d}}\right)}^{2},\\ =\frac{1}{2}{\left\|S^{\text{d}}-B^{\text{d}}\right\|}_{2}^{2}, \end{array}$$
   where *S*^d^ is the normal result worth of the d-th test, and *B*^d^ addresses the genuine result worth of the d-th test after the organization activity.
(b) Backpropagation
The data are resolved layer by layer in the association, and the error between the veritable outcome and the ordinary outcome is obtained, which can be seen as the attention to the neuron base. Its equation is
  (2) $$\begin{array}{c} \frac{\partial E}{\partial P}=\frac{\partial E}{\partial W}\frac{\partial W}{\partial P}. \end{array}$$
The recipe for the responsiveness of layer *x* in the backpropagation stage is:
  (3) $$\begin{array}{c} \delta^{s}={\left(T^{x+1}\right)}^{S}\delta^{x+1}•g^{\prime }\left(W^{s}\right). \end{array}$$
The responsiveness of the result layer hub is
  (4) $$\begin{array}{c} {}^{\delta }=g^{\prime }\left(W^{x}\right)•\left(B^{\text{d}}-S^{\text{d}}\right). \end{array}$$
(c) Weight update
The weight update equation is
  (5) $$\begin{array}{c} \frac{\partial E}{\partial T}=P^{x-1}{\left(\delta^{x}\right)}^{S},\\ \Delta T^{x}=-\eta \frac{\partial E}{\partial T^{x}}. \end{array}$$

The particular preparation interaction of the convolutional layer is as follows:

It inputs the information to the convolution layer for convolution estimation and gets:

(6) $$\begin{array}{c} P_{n}^{x}=g\left(\sum_{m\in R_{n}}P_{m}^{x-1}•T_{mn}^{x}+L_{n}^{x}\right). \end{array}$$

As in condition 9, it is shown that the computation is the slant of the convolutional layer:

(7) $$\begin{array}{c} \delta_{n}^{x}=\beta_{n}^{x+1}\left(g^{\prime }\left(W_{n}^{x}\right)•\text{up}\left(\delta_{n}^{x+1}\right)\right), \end{array}$$

where up(•) is the upsampling calculation.

Through the above computation, the given component map slope is acquired. Recipe 10 shows that the slope of the predisposition premise is found by adding the awareness of the element map hubs in layer *x*:

(8) $$\begin{array}{c} \frac{\partial E}{\partial L_{n}}=\sum_{i,j}{\left(\delta_{n}^{s}\right)}_{ij}. \end{array}$$

The inclination of the convolution piece loads is determined as follows:

(9) $$\begin{array}{c} \frac{\partial E}{\partial K_{mn}^{x}}=\text{rot}180\left(\text{conv}2\left(A_{m}^{x-1},\text{rot}180\left(\delta_{n}^{x}\right),\prime \text{valid}\prime \right)\right). \end{array}$$

Finally, the weights are updated with the above formula, and the same is true when updating the bias.

The pooling examining layer preparing process is as follows:

(10) $$\begin{array}{c} P_{n}^{x}=g\left(\beta_{n}^{x}\text{down}\left(P_{n}^{x-1}\right)+L_{n}^{x}\right), \end{array}$$

where down(•) is the pooling function, and *β* and *L* represent the weight and bias, respectively.

(11) $$\begin{array}{c} \delta_{n}^{x}=g^{\prime }\left(W_{n}^{x}\right)•\text{conv}2\left(\delta_{n}^{x+1},\text{rot}180\left(K_{n}^{x+1}\right),\prime \text{full}\prime \right). \end{array}$$

The estimation of the predisposition in the pooled examining layer is equivalent to the computation of the predisposition in the convolutional layer. Yet, the estimation recipe of weight *β* is as follows:

(12) $$\begin{array}{c} \frac{\partial E}{\partial L_{n}}=\sum_{i,j}{\left(\delta_{n}^{x}•f_{n}^{x}\right)}_{ij}, \end{array}$$

where

(13) $$\begin{array}{c} f_{n}^{x}=\text{down}\left(P_{n}^{x-1}\right). \end{array}$$

At last, the loads are refreshed by equations (12) and (13).

### 3.2. Deep Reinforcement Learning Methods

#### 3.2.1. Reinforcement Learning

As indicated by the different learning criticism components, AI calculations can be isolated into 3 classifications: directed learning, solo learning, and support learning [21, 22]. It is to solve such a problem: the agent (Agent) selects the best action by learning to achieve the preset optimal goal. Its basic framework is shown in Figure 6.

The agent in this RL process can be simplified as a state set *D* and an action set *G*. *D* contains all the states that the Agent may encounter. *G* represents the set of all possible actions to perform.

#### 3.2.2. Agent's Learning Algorithm

An Agent in a reinforcement learning system can be composed of one or more of three elements: policy, value function, and model. The policy means that the agent decides its actions according to the state at a given moment. It is a mapping relationship between states and actions. It can be in one-to-one correspondence, or it can be expressed in the form of probability, that is the probability of performing an action in a certain state. The value function represents the cumulative sum of rewards starting from the current state. Generally speaking, the value of the value function corresponding to the optimal policy is the largest [23]. The model indicates that the agent has all the knowledge of environment replacement and change, that is it can predict what the next state of the environment will be. From the perspective of a Markov decision process, it represents information about its state, action, state transition function, and reward function. According to whether elements such as strategy, value function, and model are included in the process of solving the problem, the learning algorithms of Agent can be divided into five categories as shown in Figure 7.

The *K*-learning algorithm belongs to the category of model-free learning algorithms and is a classic representative of the solution method based on the value function. It can represent its policy hypothesis $\overset{⌢}{K}$ by constructing a large table, where each state-action pair corresponds to a table item $\overset{⌢}{K}\left(D,G\right)$. Based on the current environmental state *D*, the agent chooses to perform an action *G*, and then observes the reward value *E* and the next state *D*′. The agent repeats this process until the end of the episode (Episode) and updates $\overset{⌢}{K}\left(D,G\right)$ with the below formula.

(14) $$\begin{array}{c} \overset{⌢}{K}\left(D,G\right)\leftarrow E+\gamma \underset{G^{}}{\max}\overset{⌢}{K}\left(D^{\prime },G^{\prime }\right). \end{array}$$

### 3.3. Crawler Self-Propelled Rotary Tiller Based on Deep Learning Network

The tractor automatic tillage control system is mainly composed of controller, electro-hydraulic proportional reversing valve, double-acting oil cylinder, control panel, speed measuring radar, angle sensor, tension pressure sensor, and encoder. The tractor automatic tillage depth control system mainly realizes the hydraulic suspension automatic control based on the three parameters of force-position-slip rate. It is mainly based on force level control, considering the control of slip rate [24]. The working principle of the system is shown in Figure 8.

#### 3.3.1. Structural Design and Working Principle

The design of crawler self-propelled rotary tiller consists of an engine, hydraulic and operating system, electrical system, and other parts. It uses a 74 kW name-brand engine with nominal power and is located under the front driver's seat. It can independently provide power for steering drive traveling system, hydraulic system, and main engine working device. The chassis is a crawler self-propelled structure, including a gearbox, a hydrostatic continuously variable transmission (HST), a chassis frame, a supporting wheel train, a walking track, and a control device, which are used for walking and transferring during operations [25].

The machine adopts crawler-type traveling mechanism—tractor driving principle. It adopts independent three-point suspension, and the working width of the rotary tiller is 220 cm. The power of the engine is transmitted to the driving wheel through the gearbox, and the traction force is transmitted to the ground through the rubber crawler meshed on the driving wheel, and then the crawler is driven relative to the ground through the ground reaction force. Another part of the engine power is transmitted to the rotary tiller through the belt drive and then through the rotary tiller gearbox. Ploughing and ploughing operations are carried out using the compound motion of the rotation of different blades and the advance of the crawler [26].

The design appearance and main technical parameters are shown in Figure 9 and Table 1, respectively.

#### 3.3.2. Main Technical Features

1. It adopts an 80-type gearbox, 45 displacement HST, and 340 mm ground clearance, which improves the passability and reliability of the rotary tiller during operation (as shown in Figure 10(a)).
2. It adopts lengthened and widened high-patterned crawler tracks with a size of 90 × 51 sections × 450 (mm), which has a stronger gripping ability and lower ground pressure, which improves the passability of the machine. At the same time, the new chassis structure is adopted to ensure the stability of the whole machine (as shown in Figure 10(b)).
3. The lifting height of the rotary tiller is increased to 700 mm above the ground, which improves the passability of the whole machine. The structure of double oil cylinders ensures the working stability of the rotary tiller (as shown in Figure 10(c)).
4. The round cutter roller is selected to meet the needs of paddy fields in different regions. The weed prevention has enlarged the bolt flange structure, which has high reliability and convenient maintenance. As shown in Figures 11 and 12, the transmission is side gear, the gear module is large, and the structure is reliable.
5. Using one lever operation (as shown in Figure 13), the lifting and lowering of the rotary tiller and the left and right turning of the machine are all completed with one lever, which is easy and convenient to operate. Using a hydraulic solenoid valve (as shown in Figure 14) and an HST device, walking and steering are more comfortable.
6. Adopting independent three-point suspension mode, which can realize multipurpose of one machine, suitable for paddy field and dry land. It can also be equipped with agricultural tools such as ditching, ridge, and fertilization, which improves the utilization rate of machinery and tools and increases revenue.

#### 3.3.3. Technological Innovation Points

(1) Innovation of walking mode and power output. (2) Unique design innovation of the chassis. (3) Rotary tiller cutter and anti-grass device. (4) Reasonable distribution of the walking speed and the cutting speed of the rotary tiller.

### 3.4. System Performance of Crawler Self-Propelled Rotary Tiller

#### 3.4.1. Driving Principle of Crawler Self-Propelled Rotary Tiller

Similar to the principle of wheeled running gear, in order for a crawler vehicle to travel on a level road, the following two conditions must be met:

- A driving force of sufficient magnitude to enable the drive sprocket to rotate;
- The crawler adhesion force of the grounded part of the running gear is greater than the sum of the various driving resistances.

The resistance includes operation resistance such as cutting and earthmoving, rolling resistance between the track and the road surface, and internal friction between each component and the track.

(15) $$\begin{array}{c} H_{g}=H_{j}+H_{k}+H_{l}, \end{array}$$

where *H*_*g*_ is the driving torque converted from the engine to the driving sprocket; *H*_*j*_ is the torque required to overcome the horizontal resistance; *H*_*k*_ is the moment required to overcome the rolling resistance of the track and the ground; and *H*_*l*_ is the torque required to overcome the internal friction of each component and the track.

Due to the large number of track shoes and the large grounding area, each track shoe will be subjected to the ground reaction force Δ*P*_*i*_, so the horizontal traction force of the entire track is:

(16) $$\begin{array}{c} P_{g}=\sum \Delta P_{i}. \end{array}$$

#### 3.4.2. Kinematic Analysis of Crawler Walking System

The motion of a crawler system is similar to that of a chain drive. When doing kinematic calculations, the average speed of the track winding is usually calculated using the total length of the chain links that the drive wheel has turned. The formula is as follows:

(17) $$\begin{array}{c} V_{j}=\frac{x_{0}l_{0}q_{0}}{2\pi },\\ =\frac{x_{0}l_{0}n_{0}}{60}\left(\frac{m}{s}\right), \end{array}$$

where *l*_0_ is the track pitch (m); *x*_0_ is the number of teeth of the driving wheel; *q*_0_ is the angular velocity of the driving wheel (rad/s); and *n*_0_ is the drive wheel speed (r/m).

During the driving process of the crawler self-propelled rotary tiller, if there is no relative sliding between the crawler shoe and the ground, the theoretical speed is the running speed of the crawler bulldozer, that is, when the driving wheel and the track links are driven, the average speed of the track is the running speed of the track rotation, the formula is as follows:

(18) $$\begin{array}{c} V_{r}=\frac{x_{0}l_{0}q_{0}}{2\pi },\\ =\frac{x_{0}l_{0}n_{0}}{60}\left(\frac{m}{s}\right). \end{array}$$

Or

(19) $$\begin{array}{c} V_{r}=r_{0}•q_{0}, \end{array}$$

where *r*_0_ is the pitch circle radius (m) of the driving wheel.

When the simplified kinematic analysis of the crawler-type traveling system is performed, the calculation of the traveling speed of the crawler-type machine is usually carried out according to formula (19).

When the crawler self-propelled rotary cultivator travels forward, the adhesion between the grounded part of the crawler and the ground is greater than the sum of the driving resistances, and the crawler shoe squeezes the ground in the horizontal direction to deform the soil and generate a shear resistance, so there will be slippage of the crawler, and the actual speed *v* of the crawler walking system is less than its theoretical speed *V*_*r*_, that is

(20) $$\begin{array}{c} V=V_{r}-V_{b}, \end{array}$$

where *V*_*b*_ is the slip speed of the track.

Track slippage is very small when running empty. To simplify the calculation, the no-load running speed *V*_0_ is used instead of the theoretical speed.

## 4. Experiment of Crawler Self-Propelled Rotary Tiller Driving Rice Farming Based on Deep Learning

It adopts the self-developed crawler-type rotary tiller and straw stubble pulper to conduct a comparative test on the field operation performance of the combination of common wheeled tractor and rotary tiller. A total of 3 treatments were set up in this test, namely Wode Aolong WD704F wheeled tractor + 1GZL-220 rotary tiller (B1), self-developed crawler tractor + 1GZL-220 rotary tiller (B2), and self-developed crawler tractor + self-developed straw returning pulper (B3). The number of tillage times was 2, and the previous stubble crop in the experimental field was early rice, which was harvested by a full-feed combine harvester with a crushing device, and the average stubble height was 15 cm. The area of the experimental field is 3 mu, and the field is divided into 3 plots, each with an area of 666.67 m^2^. The straw was crushed and returned to the field in full. The fields were irrigated and soaked for 2 d before the rotary tillage operation, and the irrigation depth was 50 mm.

### 4.1. Farming Effect

Table 2 shows the comparative test results of the field operation performance of the self-developed crawler-type rotary tiller + straw stubble pulper at different stubble heights. It can be seen from Table 2 at the developed paddy field rice straw returning and pulping machine in the south can complete a number of operation procedures such as returning the high stubble straw to the paddy field, rotary tillage, and surface leveling at one time. Except when the stubble height is 450 mm and the number of operations is 1 time, the stubble pressing depth is 49.5 mm, which is slightly lower than the technical requirements, the five indexes of tillage depth, tillage depth stability, stubble pressing depth, ground flatness, and vegetation coverage qualification rate of the other treatments all met the technical requirements. When tilled twice, even the highest stubble height was 450 mm, all the indicators were significantly in line with the technical requirements. It can be seen from Figure 15 that when the stubble height is 150 mm and the number of tillage times is 2, the indicators are significantly better than other treatments. The qualified rates of tillage depth, tillage depth stability, stubble depth, ground flatness, and vegetation coverage were 141.64 mm, 94.82%, 98.67 mm, 25.13 mm, and 94.60%, respectively. Compared with the national standard, it increased by 18.03%, 11.55%, 97.34%, 49.74%, and 18.25% respectively, which significantly improved the farming effect.

Table 3 shows the field performance test results of different tillage tools. From Table 3, it is clear that the exhibition marks of various culturing instruments are altogether unique. From B1 to B3, the effect of each tillage index increases sequentially. The ploughing depth, ploughing depth stability, stubble depth, ground flatness, and vegetation coverage qualification rate of the B3 treatment were 141.64 mm, 94.82%, 98.67 mm, 25.13 mm, and 94.60%, respectively, which were significantly better than the other two treatments. Compared with B1 and B2, the indicators increased by 9.92% and 4.88%, 4.31% and 4.13%, 42.59% and 19.12%, 40.15% and 34.57%, and 13.04% and 7.16% respectively.

### 4.2. Adaptability to Machine Insertion

Table 4 shows the effect of different stubble heights on the effect of machine transplanting. With the increase of the remaining stubble height, the planting depth decreased in turn, and the rate of missing and damaged seedlings increased gradually. There was no significant difference in the rate of drifting, and the number of tillage also affected the effect of transplanting. When the number of tillage times is 2, the effect is significantly better than that of 1-time tillage. When the number of tillage times was 1, the rate of damaged seedlings increased significantly. The self-developed crawler tractor + self-developed straw returning pulper for farming, except that the seedling damage rate does not meet the standard requirements, all indicators meet the requirements. The best results are obtained with H1N2. The planting depth, missed planting rate, floating seedling rate, and seedling injury rate of each index were 37.30 mm, 0.6%, 1.2%, and 1.2%, respectively, which were significantly better than other treatments.

Table 5 shows the effect of different tillage tools on the effect of machine transplanting. The effects of different tillage tools on the effect of machine transplanting are significantly different except for the planting depth. From B1 to B3, the pace of missing seedlings, the pace of drifting seedlings, and the pace of harmed seedlings diminished thus. The establishing profundity, the pace of missing seedlings, the pace of floating seedlings, and the pace of harmed seedlings of the B3 treatment were fundamentally better compared to those of different medicines.

### 4.3. Influence on Yield and Composition Factors

Table 6 shows the effects of different stubble heights on yield and composition factors. With the increment of stubble level, the number of compelling panicles, the number of grains per panicle, and the seed setting rate diminished progressively, and the distinction in 1000-grain weight was not huge. The number of tillage also affects the yield structure of rice. Thousand kernel weight and seed setting rate were not significantly different. The effect of the H1N2 treatment was the best, the effective panicle number reached 409.85 × 104 panicle.hm^−2^, and the number of grains per panicle reached 144.12. The theoretical yield and actual yield reached 10186.21 kg·hm^−2^ and 7115.55 kg·hm^−2^, respectively, and the yield increase effect was significant.

Table 7 shows the effects of different tillage tools on yield and composition factors. From B1 to B3, the effective panicle number, grain number per panicle, theoretical yield, and actual yield increased sequentially. The effect of the B3 treatment was significantly better than other treatments, but the difference in 1000-grain weight and seed setting rate was not significant [27, 28].

Table 8 is a comparison of the yield-increasing effect of the actual yield of different tillage tools. The B3 treatment has a significant effect on increasing production. Compared with B1 and B2, the average yield increased by 625.35 kg·hm^−2^ and 310.95 kg·hm^−2^, respectively, with an average yield increase rate of 9.63% and 4.57%.

## 5. Discussion

In one operation, the operation performance meets the technical requirements of relevant standards. When the operation is performed twice, all technical requirements fully meet the design requirements and the technical requirements of relevant standards. Compared with the national standard, it has increased by 18.03%, 11.55%, 97.34%, 49.74%, and 18.25% respectively. The operation process is stable, and the rotary tillage and surface leveling are of good quality.

The effect of straw burying and returning to the field is good. After returning the high stubble straw to the paddy field in the south, the pulping machine has a good effect on the quality of the machine. When the number of tillage times was 1, all the indicators met the requirements except the rate of damaged seedlings which did not meet the standard requirements. When the number of tillage times is 2, the performance indicators of each machine planting meet the requirements of national standards and the agronomic requirements for subsequent rice planting. The planting depth, missed planting rate, floating seedling rate, and seedling injury rate of each index were 37.30 mm, 0.6%, 1.2%, and 1.2%, respectively, which were significantly better than other treatments.

Through the performance test results of different tillage tools, it is shown that the self-developed crawler self-propelled tractor is used with the self-developed paddy field straw returning pulper to have a significant effect. Compared with wheeled tractor + ordinary rotary tiller and self-developed crawler tractor + ordinary rotary tiller, the tillage performance indicators such as working depth, tillage depth stability, ground flatness, stubble pressing depth, and vegetation coverage qualification rate are improved by 9.92% and 4.88%, 4.31% and 4.13%, 42.59% and 19.12%, 40.15% and 34.57%, and 13.04% and 7.16%, respectively. The machine transplanting indexes such as the planting depth, the rate of missing planting, the rate of drifting seedlings, and the rate of damaged seedlings were all significantly better than those of other treatments. The field test showed a significant increase in yield, with an average yield increase of 625.35 kg·hm^−2^ and 310.95 kg·hm^−2^ and with an average yield increase rate of 9.63% and 4.57%, respectively. Compared with the traditional tillage tools, the self-developed crawler self-propelled tractor + the self-developed paddy field returning pulper has a remarkable effect, which is suitable for promotion and application in the southern double-cropping rice area.

## 6. Conclusions

This article studies a conservation tillage mode of paddy field in southern China with “crawler self-propelled tractor + straw stubble pulper.” This mode can complete arable land leveling and straw returning operations at one time. Field performance tests show that the tillage performance indicators such as the working depth, tillage depth stability, ground flatness, stubble pressing depth, and vegetation coverage qualification rate of the “crawler self-propelled tractor + straw stubble pulper” are better than those of “wheel tractor + ordinary rotary tiller” and “crawler tractor + ordinary rotary tiller,” increased by 9.92% and 4.88%, 4.31% and 4.13%, 42.59% and 19.12%, 40.15% and 34.57%, and 13.04% and 7.16%, respectively. The mechanical transplanting index was significantly better than other treatments. The yield increase effect of the field test is remarkable, with the average yield increase rate of 9.63% and 4.57%, which is suitable for popularization and application in the southern double-cropping rice area.

## Figures and Tables

**Figure 1:** Schematic diagram of deep learning.

**Figure 2:** Autoencoder training flowchart.

**Figure 3:** Structure diagram of restricted Boltzmann machine.

**Figure 4:** The logistic regression step function formula.

**Figure 5:** An illustration of a convolutional brain organization.

**Figure 6:** The basic framework of reinforcement learning.

**Figure 7:** Classification of Agent learning methods.

**Figure 8:** The working principle of the tractor's automatic tillage depth control system.

**Figure 9:** Crawler self-propelled rotary tiller.

**Figure 10:** Structural features of crawler self-propelled rotary tiller. (a) Ground clearance. (b) Tracks. (c) Ground clearance.

**Figure 11:** Knife roll.

**Figure 12:** Side gear.

**Figure 13:** Joystick figure.

**Figure 14:** Hydraulic solenoid valve.

**Figure 15:** Comparison with the national standard after farming twice.

**Table 1:** Main technical parameters.

Serial number	Project		Unit	Design value
1	Specification and model		—	1GZL-220
2	Overall dimension (length × wide × high)		mm	4000 × 2500 × 2860
3	Overall quality		kg	2125
4	Hourly productivity		hm^2^/h	0.24∼0.40
5	Gauge		mm	1200
6	Minimum ground clearance		mm	340
7	Operation speed		kg/h	0∼0.58
8	Track pitch		mm	90
9	Number of track joints		Festival	51
10	Track width		mm	450
11	Maximum driving speed		kg/h	8.3
12	PTO speed		r/min	580
13	Fuel consumption		kg/hm^2^	≤15
14	Minimum ground clearance		mm	330
15	Engine	Structural style	—	In line, water-cooled, 4-stroke, direct injection turbocharging
16		Calibration power	kW	74
17		Calibration speed	r/min	2600
18	Rotary tillage part	Operation width	mm	2200
19		Ploughing depth	cm	Dry land: ≥12; paddy field ≥10
20		Number of rotary tillage knives	Handful	68
21		Rotary tiller model	—	IT245
22		Rotating speed of rotary tillage knife roller	r/min	280∼330

**Table 2:** Test results of field performance with different stubble heights.

Handle	Ploughing depth (mm)	Tillage depth stability (%)	Stubble depth (mm)	Surface flatness (mm)	Vegetation coverage (%)
H1N1	132.27c	88.79b	60.13d	44.13b	86.66b
H2N1	124.18d	86.13c	54.50e	45.94b	83.57c
H3N1	123.73d	85.45c	49.50f	48.76a	81.35d
H1N2	141.64a	94.82a	98.67a	25.13e	94.60a
H2N2	140.05a	90.56b	88.67b	34.42d	87.93b
H3N2	138.36b	89.15b	74.50c	41.64c	83.20c

**Table 3:** Field performance test results of different tillage tools.

Handle	Ploughing depth (mm)	Tillage depth stability (%)	Stubble depth (mm)	Surface flatness (mm)	Vegetation coverage (%)
B1	128.86 c	90.90c	69.20c	41.99a	83.69c
B2	135.05 b	91.06b	82.83b	38.41b	88.28b
B3	141.64a	94.82a	98.67a	25.13c	94.60a

**Table 4:** Effects of different stubble heights on the effect of machine transplanting.

Handle	Planting depth (mm)	Missing insertion rate (%)	Floating seedling rate (%)	Seedling injury rate (%)
H1N1	35.50b	1.0c	2.0bc	2.4d
H2N1	27.00e	1.2b	2.4b	6.4b
H3N1	22.50f	2.6a	3.2a	8.4a
H1N2	37.30a	0.6c	1.2cd	1.2e
H2N2	32.95c	1.4b	1.4c	4.6c
H3N2	30.25d	1.4b	2.4b	5.4bc

**Table 5:** Effects of different tillage tools on the effect of machine transplanting.

Handle	Planting depth (mm)	Missing insertion rate (%)	Floating seedling rate (%)	Seedling injury rate (%)
B1	43.20a	2.6a	2.4a	3.6a
B2	35.30c	2.4a	1.8b	2.8b
B3	37.30b	0.6b	1.2c	1.2c

**Table 6:** Effects of different stubble heights on yield structure.

Handle	Effective panicle (10^4^·hm^−2^)	Number of grains per panicle	1000-grain weight (g)	Seed setting rate (%)	Theoretical yield (kg·hm^−2^)	Actual output (kg·hm^−2^)
H1N1	387.57b	142.22ab	21.38a	80.36a	9470.91b	6618.53c
H2N1	366.06d	139.98bc	21.31b	79.73ab	8706.18d	6340.05d
H3N1	361.41d	139.09bc	21.24c	78.72ab	8404.59e	6169.87e
H1N2	409.85a	144.12a	21.34a	80.81a	10186.21a	7115.55a
H2N2	382.29b	143.36a	21.36a	80.34a	9405.27b	6827.18b
H3N2	374.43c	140.13b	21.37a	79.69ab	8935.02c	6519.37c

**Table 7:** Effects of different tillage implements on yield structure.

Handle	Effective panicle (10^4^·hm^−2^)	Number of grains per panicle	1000-grain weight (g)	Seed setting rate (%)	Theoretical yield (kg·hm^−2^)	Actual output (kg·hm^−2^)
B1	388.76c	141.13b	21.28a	78.51a	9166.68c	6490.20c
B2	391.82b	142.75b	21.32a	79.38a	9466.73b	6804.60b
B3	409.85a	144.12a	21.34a	80.81a	10186.21a	7115.55a

**Table 8:** Comparison of yield-increasing effects of different tillage implements.

Handle	Actual output (kg·hm^−2^)	B3 is higher than B1		B3 is higher than B2	
		kg·hm^−2^	%	kg·hm^−2^	%
B1	6490.20	625.35	9.63	310.95	4.57
B2	6804.60				
B3	7115.55				

## Data Availability

No data were used to support this study.
